The article "Demonstration of Cross-Protective Vaccine Immunity against an Emerging Pathogenic Ebolavirus Species" was published in 2010. Journal: PLoS Pathog.

# Demonstration of Cross-Protective Vaccine Immunity against an Emerging Pathogenic Ebolavirus Species

**DOI:** 10.1371/journal.ppat.1000904

**Published:** 2010-05-20

**Authors:** Lisa E. Hensley, Sabue Mulangu, Clement Asiedu, Joshua Johnson, Anna N. Honko, Daphne Stanley, Giulia Fabozzi, Stuart T. Nichol, Thomas G. Ksiazek, Pierre E. Rollin, Victoria Wahl-Jensen, Michael Bailey, Peter B. Jahrling, Mario Roederer, Richard A. Koup, Nancy J. Sullivan

**Affiliations:** 1 Virology Division, United States Army Medical Research Institute of Infectious Diseases, Fort Detrick, Maryland, United States of America; 2 Biodefense Research Section, Vaccine Research Center, National Institute of Allergy and Infectious Disease, National Institutes of Health, Bethesda, Maryland, United States of America; 3 Special Pathogens Branch, Division of Viral and Rickettsial Diseases, Centers for Disease Control and Prevention, Atlanta, Georgia, United States of America; 4 Integrated Research Facility, National Institute of Allergy and Infectious Diseases, National Institutes of Health, Bethesda, Maryland, United States of America; 5 Immunology Laboratory, Vaccine Research Center, National Institute of Allergy and Infectious Disease, National Institutes of Health, Bethesda, Maryland, United States of America; Mount Sinai School of Medicine, United States of America

## Abstract

A major challenge in developing vaccines for emerging pathogens is their continued evolution and ability to escape human immunity. Therefore, an important goal of vaccine research is to advance vaccine candidates with sufficient breadth to respond to new outbreaks of previously undetected viruses. Ebolavirus (EBOV) vaccines have demonstrated protection against EBOV infection in nonhuman primates (NHP) and show promise in human clinical trials but immune protection occurs only with vaccines whose antigens are matched to the infectious challenge species. A 2007 hemorrhagic fever outbreak in Uganda demonstrated the existence of a new EBOV species, Bundibugyo (BEBOV), that differed from viruses covered by current vaccine candidates by up to 43% in genome sequence. To address the question of whether cross-protective immunity can be generated against this novel species, cynomolgus macaques were immunized with DNA/rAd5 vaccines expressing ZEBOV and SEBOV glycoprotein (GP) prior to lethal challenge with BEBOV. Vaccinated subjects developed robust, antigen-specific humoral and cellular immune responses against the GP from ZEBOV as well as cellular immunity against BEBOV GP, and immunized macaques were uniformly protected against lethal challenge with BEBOV. This report provides the first demonstration of vaccine-induced protective immunity against challenge with a heterologous EBOV species, and shows that Ebola vaccines capable of eliciting potent cellular immunity may provide the best strategy for eliciting cross-protection against newly emerging heterologous EBOV species.

The article "Demonstration of Cross-Protective Vaccine Immunity against an Emerging Pathogenic Ebolavirus Species" was published in 2010. Journal: PLoS Pathog.

## Author Summary

Ebola virus causes death, fear, and economic disruption during outbreaks. It is a concern worldwide as a natural pathogen and a bioterrorism agent, and has caused death to residents and tourists of Africa where the virus circulates. A vaccine strategy to protect against all circulating Ebola viruses is complicated by the fact that there are five different virus species, and individual vaccines provide protection only against those included in the vaccine. Making broad vaccines that contain multiple components is complicated, expensive, and poses challenges for regulatory approval. Therefore, in the present work, we examined whether a prime-boost immunization strategy with a vaccine targeted to one Ebola virus species could cross protect against a different species. We found that genetic immunization with vectors expressing the Ebola virus glycoprotein from Zaire blocked infection with a newly emerged virus species, Bundibugyo EBOV, not represented in the vaccine. Protection occurred in the absence of antibodies against the second species and was mediated instead by cellular immune responses. Therefore, single-component vaccines may be improved to protect against multiple Ebola viruses if they are designed to generate this type of immunity.

## Introduction

The *Ebolavirus* genus of the family *Filoviridae* was thought previously to consist of four species, ZEBOV, SEBOV, Reston (REBOV), and Cote d'Ivoire (CIEBOV) [1]. Of these, ZEBOV and SEBOV have been associated with the majority of Ebola virus hemorrhagic fever (EHF) cases in humans [2]. Within the last decade, the frequency of EBOV outbreaks in Africa has increased, probably due to human encroachment on the natural habitat of animal reservoir(s) and/or improved surveillance [3]. Due to the aggressive nature of EHF symptoms, the rapid spread of infection to other persons in close contact with the infected individual, resultant high mortality rate and threat of bioterrorism, vaccine development against EBOV virus is a high priority. EHF vaccines based on recombinant adenovirus serotype 5 (rAd5) vectors encoding the ZEBOV and SEBOV envelope glycoproteins, GP(Z) and GP(S/G), respectively, have shown protective efficacy in NHP [4], [5], [6] and hold promise as vaccine candidates for human use [7]. In addition to rAd vaccines, other viral-vectored and virus-like particle (VLP) vaccines have exhibited protective efficacy against EBOV infection in NHP [8], [9], [10]. Though each of these vaccines generates potent immune responses in NHP, protection is achieved only when the vaccine immunogen and the EBOV species used for infectious challenge are matched, and data show a lack of cross protection against antigens not contained in the vaccine [8], suggesting that existing vaccines may not provide coverage against newly emerging EBOV species.

The article "Demonstration of Cross-Protective Vaccine Immunity against an Emerging Pathogenic Ebolavirus Species" was published in 2010. Journal: PLoS Pathog.

An outbreak of HF in Western Uganda in late 2007 led to the identification of a fifth species in the genus *Ebolavirus* [11]. Complete genome sequence comparison of all EBOV species revealed that the virus from Western Uganda, the Bundibugyo species, differed from the previously characterized four EBOV species by 32–42%, as is characteristic for divergence between other members in the genus. Current human vaccine candidates encode GP from SEBOV and ZEBOV, whose sequences differ from BEBOV by 38–47% at the amino acid level. The lack of cross protection of existing vaccines against heterologous species with sequence divergence in the same range suggests that vaccines currently in development will not protect against emerging Ebola viruses. We have shown previously that a prime-boost vaccine strategy priming with DNA vectors and using rAd vectors to provide the boost generates broad immune responses across both T- and B-cell immune compartments [6]. This immunization regimen has been demonstrated to generate antigen-specific immune responses at least one log higher than those observed with either DNA or rAd alone [12]. Therefore, we hypothesized that a DNA prime/rAd5 EBOV vaccine strategy would be the most likely candidate to induce cross-protection against BEBOV. We demonstrate herein that potent responses induced by prime-boost vaccination can provide immune protection against newly emerging EBOV species and show for the first time vaccine-induced species cross-protection against EBOV infection.

## Results

### Immunization of cynomolgus macaques with DNA/rAd

It has been demonstrated previously that NHP immunized with a vaccine consisting of EBOV GP DNA followed by boosting with rAd5 GP were uniformly protected when challenged with a lethal dose of wild-type ZEBOV, Mayinga strain [6]. Four cynomolgus macaques were injected at 4–6 week intervals with GP(Z) and GP(S/G) DNA, followed by a rest period, and boosted after one year with rAd5 vectors containing the EBOV matched insert according to the schedule depicted in Figure 1A. Although sequence divergence between genes coding for BEBOV GP and the inserts contained within the previously used vaccine is substantial, homology is displayed within the N- and C-terminal regions of GP that contain structural elements critical for virus replication [13]. This genetic relatedness between species was the basis for selection of vaccine inserts with the goal of broad coverage against multiple species. Phylogenetic analysis demonstrates that ZEBOV shares genetic ancestry with CIEBOV and BEBOV, while SEBOV is closest to REBOV (Figure 1B). To assess whether ZEBOV and SEBOV gene inserts were likely to provide cross protection against heterologous infectious challenge with BEBOV, GP antigen-specific immune responses in humoral and T cell compartments were assessed by ELISA and intracellular cytokine staining (ICS), respectively, three weeks after delivery of the rAd5-GP(Z) boost immunization.

The article "Demonstration of Cross-Protective Vaccine Immunity against an Emerging Pathogenic Ebolavirus Species" was published in 2010. Journal: PLoS Pathog.

**Figure 1:** Vaccination and challenge schedule. (A) Vaccine group NHP were injected with plasmid DNA and rAd5 vectors encoding GP from SEBOV and/or ZEBOV. Individual DNA immunizations were spaced by 4–6 week intervals and the rAd boost was given one year after the final DNA prime. Animals were exposed to a lethal dose of BEBOV 7 weeks after the rAd5 GP boost. (B) Distance matrix-based phylogenetic tree for EBOV GP. Numbers at the nodes are boostrap percentages. Vertical branches are for graphic representation; horizontal branch lengths are measured as substitutions per site (scale bar  = 0.07). The infectious challenge species is shown in blue. Vaccine strains are indicated in bold.

### Humoral immune responses elicited by prime-boost immunization

Studies performed previously have shown an absence of neutralizing antibody in vaccinated macaques and a lack of correlation with protection from infection [14], [15]. In contrast, there is a strong association between GP-specific ELISA IgG titers in serum or plasma of immunized animals and protection from EBOV infection in NHP [6], and subsequent analysis has illustrated that vaccine-induced ELISA titers correlate with protection by rAd5 based vaccines [16]. Therefore, to assess DNA/rAd vaccine immunogenicity in the current study, anti-GP ELISA IgG responses specific for the ZEBOV vaccine insert were measured at the end of the rest period following DNA immunization (pre-boost) and compared to ELISA IgG titers after boosting with rAd5-GP (post-boost)(Figure 2A). DNA priming alone induced modest plasma antibody titers, averaging an effective concentration (EC90) of 1/900 for all subjects in the vaccine group. Subsequent immunization with rAd5-GP boosted plasma titers by at least an order of magnitude in all subjects (p = 0.02, pre-boost *vs*. post-boost titers) and by two logs in subject V2. These data confirm the potency of the prime boost vaccine regimen and demonstrate that significant boosting of DNA-primed humoral immunity can be achieved even one year after the final priming immunization.

The article "Demonstration of Cross-Protective Vaccine Immunity against an Emerging Pathogenic Ebolavirus Species" was published in 2010. Journal: PLoS Pathog.

**Figure 2:** Development of vaccine-induced antibody responses. (A) The quantity of anti-Ebola GP IgG in plasma samples from vaccinated cynomolgus macaques was determined by ELISA as described in Methods. Results are shown for samples obtained after the final DNA prime and prior to immunization with rAd (pre-boost, light blue), and for samples obtained 3 weeks after boosting with rAd-GP (post-boost, dark blue). Plasma antibody titers are presented as EC90 reciprocal dilution titers. (B) ELISA IgG against ZEBOV (blue) and BEBOV (red) antigens. Plasma dilution series are shown for each immunized subject. The averages for negative control samples (n = 4) are shown for ZEBOV (black dotted line) and BEBOV (black dashed line).

As an initial assessment of potential vaccine-induced cross-species immunity against BEBOV, subject plasma samples were evaluated using the same ELISA format described above except the capture antigen used was BEBOV GP. Comparison of subject antibody responses against BEBOV and ZEBOV (Figure 2B) shows that the ZEBOV DNA/rAd vaccine did not generate antibodies cross-reactive with BEBOV GP. Anti-BEBOV reactivity for all four vaccine subjects overlapped the average background level of antigen binding displayed by samples from unvaccinated control subjects (n = 4). The absence of cross-specific antibody reactivity suggests that immunoglobulins elicited by the DNA/rAd vaccine were directed against linear amino acid sequences not contained within BEBOV GP or against conformational epitopes dependent on protein tertiary structure.

### Vaccine induction of cross-reactive CD4^+^ and CD8^+^ T cells

In earlier work, DNA/rAd5 vaccine-induced EBOV cellular immunity was assessed by measuring *in vitro* antigen-activated cell proliferation in PBMC obtained from immunized subjects. While proliferation assays provide a useful measure of T-cell immunity, important effector cell activity, especially within the CD8 T-cell compartment, may not be captured in these measurements [17]. Therefore, we evaluated PBMC from immunized macaques using intracellular cytokine staining to assess memory and effector CD4^+^ and CD8^+^ T-cell functions. PBMC samples collected from vaccinated animals four weeks after the rAd5 GP vaccine boost were isolated by density gradient centrifugation and stimulated with peptides spanning the ZEBOV or BEBOV GP reading frame. Intracellular expression of TNFα, IFNγ, and IL-2 induced in the CD8^+^ and CD4^+^ memory T cell subsets was evaluated in PBMC samples and quantified after gating on CD95 and CD45RA memory markers (Figure 3A). DNA/rAd prime-boost EBOV immunization generated antigen-specific CD4^+^ T cell immunity against proteins expressed by the vaccine insert (Figure 3B). The magnitude of antigen-specific CD4^+^ T cells was uniform across the four immunized macaques and exceeded that observed with a single-shot rAd vaccine [5], [12], [18], [19], [20], [21], demonstrating the potency of DNA priming for augmentation of CD4^+^ T cell immunity seen by others [18]. In contrast to the species specificity demonstrated for antibody responses in this study, CD4^+^ T cells elicited by the vaccine gene inserts were cross-reactive with BEBOV GP. Intracellular cytokine secretion was stimulated by BEBOV GP in each of the vaccinated macaques, suggesting that dominant T-cell epitopes are contained within the few highly conserved GP regions of sufficient length (10–12 residues) for MHC class II presentation and TCR recognition.

The article "Demonstration of Cross-Protective Vaccine Immunity against an Emerging Pathogenic Ebolavirus Species" was published in 2010. Journal: PLoS Pathog.

**Figure 3:** T-cell immune responses measured by intracellular cytokine staining. PBMC were stimulated with overlapping peptides spanning the GP protein, and antigen-specific CD4^+^ and CD8^+^ cells were enumerated in the memory cell gates (A) by the detection of cytokine production. The percentages of cytokine-positive CD4^+^ (panel B) and CD8^+^ (panel C) T cell memory cells specific for ZEBOV (blue) and BEBOV (red) were determined at 4 weeks post rAd-GP boost. Responses are shown for each individual cytokine measured as the total proportion of cells positive for TNFα (blue), IFNγ (gray), IL-2 (red), expressed as a percentage of the memory cell population after background subtraction of control, unstimulated, samples run in parallel.

Overall, the composite cellular immune response elicited by the prime-boost immunization was skewed toward CD8^+^ T cell activity (Figure 3C). For ZEBOV, GP activation of CD8^+^ T cells was several fold higher (p = .05) than the corresponding CD4^+^ T cell responses as a percentage of the lineage memory population. Subject A01088 was a notable outlier whose CD8^+^ T responses were markedly lower than in other subjects. As observed for CD4-based immunity, CD8^+^ memory cell cytokine responses were higher than those obtained with a rAd-only vaccine, and the results showed overall that prime-boost immunization with DNA/rAd5 elicited potent antigen-specific humoral and cellular immunity. Examination of the proportions of single-, double-, and triple-positive cytokine producing cells did not reveal a dominant phenotype among the vaccinated subjects. However, the distribution of responses represented by each cytokine revealed that IL-2 positive cells were a minor component of the overall CD8^+^ T-cell responses, but contributed a greater proportion of the overall CD4+ T cell response as expected for this population which must be fit to undergo proliferation in response to pathogen exposure.

The article "Demonstration of Cross-Protective Vaccine Immunity against an Emerging Pathogenic Ebolavirus Species" was published in 2010. Journal: PLoS Pathog.

### Infectious challenge of NHP with Bundibugyo EBOV

DNA/rAd5 immunization of cynomolgus macaques protects against infection when animals are challenged with a virus species homologous to the vaccine inserts. Although there was no serological cross-reactivity between ZEBOV and BEBOV species, sequence alignment demonstrated several regions of sequence identity sufficient to comprise conserved CD4^+^ and CD8^+^ T-cell epitopes (not shown), and immunized macaques exhibited robust cellular immunity against the GP from both species. To test whether immunity was sufficiently conserved to provide protection against heterologous virus infection, ZEBOV-immunized animals were challenged with a lethal dose (1000 TCID_50_) of BEBOV. Infection was monitored using traditional measures of filovirus infection including the appearance of maculopapular rash and damage to hepatocytes [22]. The effect of infection on hepatocytes was evaluated by measuring the liver enzymes AST and ALT. By day 10 post-infection, all control subjects exhibited severe maculopapular rash (not shown) and elevated liver enzymes, and viral RNA (Figure 4), characteristic of filovirus infection in macaques. In the case of control subject C1, AST and ALT subsequently decreased to normal and near normal levels, respectively (Figure 4A,B). Three out of the four control animals succumbed to infection with BEBOV between days 12 and 13 (Figure 4D). One unvaccinated control animal (C3) survived challenge but exhibited the full constellation of EHF symptoms, suggesting that this animal was infected but successfully cleared the infection. The time course for lethal infection of control animals was somewhat longer than a comparative infectious challenge with ZEBOV which causes death in cynomolgus macaques on average within one week following challenge [23]. Among the vaccinated animals, AST levels remained normal or near normal at all tested time points (Figure 4B). Subject V4 exhibited a mild, transient increase in the serum levels of ALT, which was lower in magnitude than that observed in the control animals. Additionally, viral RNA was detected in this subject on day 6 post infection and returned to undetectable levels by the next blood draw on day 10 (Figure 4C). Thus, the four macaques that received the DNA prime/rAd5 GP boost vaccine regimen generated immunity sufficient to prevent or control BEBOV infection (p = 0.04 vs. controls). These data demonstrate that a DNA/rAd5 vaccine containing ZEBOV and SEBOV antigens provides cross-protective immunity against heterologous challenge with BEBOV.

The article "Demonstration of Cross-Protective Vaccine Immunity against an Emerging Pathogenic Ebolavirus Species" was published in 2010. Journal: PLoS Pathog.

**Figure 4:** Bundibugyo EBOV challenge. Control and vaccinated animals were exposed to a target dose of ∼1,000 TCID_50_ of BEBOV. Blood samples were collected before and after infection for the determination of hepatic enzyme levels. ALT (panel A) and AST (panel B) were measured using a General chemistry 12 reagent disk for the Piccolo Analyzer (Abaxis). Viral load (panel C) was determined by quantitative RT-PCR of plasma RNA using primers specific for BEBOV. Control and vaccinated animal values are shown in red and blue bars, respectively. Kaplan Meier survival curves (panel D) were drawn using GraphPad Prism.

## Discussion

Until recently, there were four known species of EBOV, with the most virulent being the ZEBOV and SEBOV species [24], [25]. While there is evidence pointing to fruit bats as a possible natural reservoir for EBOV, this has not yet been definitively proven. Therefore, it is difficult to successfully implement public health measures to prevent EHF outbreaks, and the potential use of EBOV as a weapon of bioterrorism also necessitates the development of medical countermeasures to prevent and/or treat infection. The absence of effective therapies to mitigate EHF symptoms and mortality reinforces the urgent need to develop an effective vaccine against EBOV. Prior studies [5], [6] demonstrated that rAd or DNA/rAd genetic vaccines against ZEBOV provide protection against challenge with an otherwise lethal dose of the homologous virus species. Towner, et al., described a fifth Ebola species in 2008, BEBOV, which was responsible for a hemorrhagic fever outbreak in Uganda with a case fatality rate of approximately 36% [11]. The Bundibugyo species has 63%, 58% and 68% sequence similarity to ZEBOV, SEBOV and CIEBOV species, respectively, and there is little serological cross reactivity between most species [26]. Since all vaccines shown to protect NHP are targeted to ZEBOV and SEBOV, it is important to determine whether new species should be incorporated as additional components of vaccine formulations against EBOV or if current vaccines may provide adequate coverage against emerging viruses such as BEBOV.

The data presented here demonstrate that a vaccination strategy targeting structural proteins from ZEBOV and SEBOV was able to provide cross-protective immunity against infectious challenge with a heterologous EBOV species. This may have been due in part to the ability of DNA/rAd prime-boost vaccination to generate more robust immune responses than single-shot vaccines. The time to death for the BEBOV controls (12–14 days) was somewhat longer than what we have observed for ZEBOV (6–12 days) [5] suggesting it may also be possible that BEBOV is less pathogenic than other EBOV species and therefore inherently more sensitive to host immunity.

The article "Demonstration of Cross-Protective Vaccine Immunity against an Emerging Pathogenic Ebolavirus Species" was published in 2010. Journal: PLoS Pathog.

The observed 100% protection against BEBOV infection in NHP would not be predicted given the divergence in GP sequence between BEBOV GP and the vaccine inserts but suggests that sufficient conservation of immunogenic regions exists between the different species. Immunization with rAd-GP one year after the final DNA prime boosted antigen-specific antibody responses to an average titer of 1/40,000 which is an order of magnitude higher than the titer predicted to correlate with survival from challenge with homologous virus, and demonstrates both potency and durability for this vaccine platform. It is noteworthy that rAd vectors demonstrated efficient boosting of the antigen-specific immune response when administered even a year after the final DNA prime. This result is not altogether surprising since it has been reported previously that longer prime-boost intervals may actually enhance immune responses induced by the boosting immunization [27], possibly because memory cells have had sufficient time to undergo complete contraction and development of a central memory phenotype. The strong boosting effect of rAd5 vectors in DNA primed subjects may also help to overcome the reduced potency of these vectors when administered to subjects with pre-existing immunity to the vaccine vector. The ability of prime-boost vaccination to generate cellular responses in the form of CD4^+^ T-cell help as well as CD8^+^ T-cell effector immunity likely accounts for the protection observed after challenge with BEBOV, since vaccinated macaques in the present study lacked antibodies reactive with BEBOV but were fully protected against disease. Although the anti GP immunoglobulins did not cross-react with BEBOV, the presence of high-titer antibodies is indicative of strong underlying antigen-specific immunity induced by the vaccine, comprising antibody, CD4^+^ and CD8^+^ T-cell functions. DNA immunization has been shown to elicit antigen-specific immunity biased toward the generation of CD4^+^ T-cell memory responses that are necessary for long term memory and potentiate CD8^+^ T-cell functions, while rAd5 vaccine boosting elicits strong antibody and CD8^+^ T-cell responses [28]. The high magnitude of CD8^+^ T-cell activity exhibited here is consistent with those findings and suggests an important role for this T-cell subset in the observed protective immunity. It is noteworthy that the animal with the lowest CD8^+^ T-cell response, V4, exhibited a transient increase in clinical markers of disease. T-cell-mediated protection from EBOV infection is supported not only by the robust CD4 and CD8 responses generated by the DNA/rAd vaccine but also by previous experiments demonstrating that passive transfer of anti-Ebola neutralizing monoclonal antibody (KZ52) into naïve rhesus macaques had no significant effect on survival when the recipients were exposed to a lethal dose of ZEBOV [15].

The article "Demonstration of Cross-Protective Vaccine Immunity against an Emerging Pathogenic Ebolavirus Species" was published in 2010. Journal: PLoS Pathog.

The findings reported herein demonstrate a mechanistic basis for vaccine-induced immune protection against EBOV infection and will therefore inform the design of next-generation vaccines. Furthermore, this study shows that it is possible to protect against EBOV species whose antigens are not present in the vaccine formulation. This suggests that current vaccines capable of eliciting robust T-cell immunity will have the greatest potential to protect against other newly emerging pathogenic EBOV species.

## Materials and Methods

### Vaccines

The vaccine vectors used in this study have been described previously [6]. Replication-defective rAd5 GP vectors were cloned and purified as described previously [29].

### Animal study and safety

Eight 3–5 year old cynomolgus macaques (Macaca fascicularis) weighing between 2–3 kg were obtained from Covance for this immunization and challenge study. All animal experiments were conducted under protocols approved by NIH and USAMRIID Animal Care and Use committees. All experiments involving the use of BEBOV in animals were performed in USAMRIID's BSL-4 laboratory. Research was conducted in compliance with the Animal Welfare Act and other federal statutes and regulations relating to animals and experiments involving animals and adheres to principles stated in the *Guide for the Care and Use of Laboratory Animals*, National Research Council, 1996. The facility where this research was conducted is fully accredited by the Association for Assessment and Accreditation of Laboratory Animal Care International. Animals were housed individually, and given enrichment regularly as recommended by the Guide for the Care and Use of Laboratory Animals (DHEW number NIH 86–23). Subjects were anesthetized with ketamine prior to blood sampling or vaccination. The vaccine and control groups each contained four cynomolgus macaques. After immunization, all the animals were transferred to the Maximum Containment Laboratory (BSL-4) at Ft. Detrick, MD for infection with BEBOV, and remained there through study completion. The monkeys were fed and checked at least daily according to the protocol.

### Macaque immunization and infection

DNA immunizations were administered by Biojector IM injection, bilateral deltoid, with a mixture of 2 mg each of two plasmid vectors encoding GP(Z) and GP(S/G). DNA immunizations were administered at 0, 4, 8, and 14 weeks. Each subject received a boost with 10^11^ particle units (PU) of rAd5 GP(Z) at 12 months following the final DNA priming immunization. All animals were challenged by the intramuscular route with 1,000 TCID_50_ of BEBOV, 7 weeks post rAd5 GP boost. The challenge virus used in this study was isolated from blood specimen #200706291 from a fatal case infected during the 2007 EBOV outbreak in Bundibugyo district, Uganda. The virus was isolated on Vero E6 cells and passaged twice prior to initiating these experiments.

The article "Demonstration of Cross-Protective Vaccine Immunity against an Emerging Pathogenic Ebolavirus Species" was published in 2010. Journal: PLoS Pathog.

### Blood chemistry

Liver enzyme levels for serum alanine aminotransferase (ALT) and aspartate aminotransferase (AST) were determined on days 0, 3, 6, 10, 14, 21 and 32 using a Piccolo Point-Of-Care blood analyzer (Abaxis, Sunnyvale, CA, USA).

### Anti-Ebola GP IgG ELISA

Methods for the GP IgG ELISA have been described previously [5]. Briefly, polyvinyl chloride ELISA plates (Dynatech, Vienna, VA, or Nunc, Rochester, NY) were coated with Ebola GP, washed, and incubated with serial dilutions of 1∶50-1∶50,000 of subject sera or plasma. Bound IgG was detected using goat anti-human IgG (H+L; Chemicon/Millipore, Billerica, MA) conjugated to horseradish peroxidase and Sigma Fast o-phenylenediamine dihydrochloride (Sigma, St.Louis, MO). The conformation-dependent antibody, KZ52, is used as a control to ensure native conformation of the capture antigen, GP. ELISA titers are expressed as effective concentration 90% (EC90) reciprocal dilution values, which represent the dilution achieving a 90% reduction in antigen binding.

### T cell intracellular cytokine secretion analysis

Peripheral blood mononuclear cells (PBMC) were isolated from cynomolgus macaque whole blood samples by separation over Ficoll, stained, and analyzed by flow cytometry essentially as described previously [4]. Briefly, PBMC were stimulated with anti-CD28 and -CD49d antibodies (BD Biosciences), Brefeldin-A (Sigma-Aldrich, St. Louis, MO), and either dimethylsulfoxide (DMSO) or a pool of 15-mer peptides overlapping by 11 spanning the ZEBOV or BEBOV GP open reading frame. Cells were stained with a mixture of antibodies against lineage markers; CD3-Cy7-APC, CD4-QD605 (BD Biosciences), CD8-TRPE, and memory markers CD95 Cy5-PE (BD Biosciences) and CD45RA QD655, fixed and permeabilized with Cytofix/Cytoperm (BD Biosciences) followed by intracellular staining with antibodies against cytokines TNFα-APC, IFNγ-Cy7-PE, and IL-2 PE. The viability dye ViViD (Invitrogen) was included to allow discrimination between live and dead cells [30]. Samples were acquired on an LSR II cytometer (BD Biosciences) and analyzed using FlowJo 8.8.5 and SPICE 5.0 software (Tree Star). Cytokine-positive cells are expressed as a percentage within CD4^+^ and CD8^+^ T cell memory subsets after subtraction of non-specific background responses that were measured in parallel for each sample.

The article "Demonstration of Cross-Protective Vaccine Immunity against an Emerging Pathogenic Ebolavirus Species" was published in 2010. Journal: PLoS Pathog.

### RNA isolation and quantitative real-time RT-PCR (qRT-PCR)

Total RNA was isolated by mixing in a ratio of 1 to 4.85 plasma sample to TRI Reagent BD (Sigma). Samples were decontaminated with 3% Lysol and then transferred from the high containment-level laboratory to a BSL3 room. RNAs was extracted with the RNAqueous kit (Ambion) and tested for BEBOV by a qRT-PCR assay. Primers and TaqMan probe for qRT-PCR were designed using the Primer Express software v2.0 (Applied Biosystem, Foster, CA). The primers/probe were: BEBOV Fw NP 5′-TGGAAACCAAGGCGAAACTG-3′; BEBOV Rv NP 5′-ACTTGTGGCATTGGCTTGTCT-3′; BEBOV Probe 5′ FAM-CCACGGGTAGCCCCCAACCAATACA- BHQ1-3′. Samples were prior tested in control PCR runs with either no RNA template or reverse transcriptase enzyme. One step qRT-PCRs were performed in triplicate using Iscript One-step RT-PCR kit (Bio-rad, Hercules, CA) in 25 µl volumes, containing 6 ng total RNA, 12.5 µM each primer, 5 µM probe and 0.25 µl reference dye BD636 (Megabase, Inc, USA). To make a standard curve for the absolute quantification, a BEBOV synthetic NP RNA was generated. The fragment was amplified from a virus containing -RNA sample with the primers BEBOV Fw NP 5′-AAACGATGGTGGGTATAATA-3′ and BEBOV Rv NP 5′-AGCGGGAGGTGCAGTGGCAGGCT-3′ and then cloned in the bidirectional transcriptional vector PCR II-TOPO (Invitrogen, Carlsbad, CA). Sequence and orientation of the cloned DNA was confirmed by sequencing reaction. After *in vitro* transcription using MAXIscript SP6/T7 Kit (Ambion), the RNA was treated with DNAse-RNAse free (Ambion), run onto 6%-urea acrylamide gel and purified by gel-excision followed by elution at 65°C for 4 hrs. For each run, a standard curve was generated from triplicate samples of dilution of the purified RNA, ranging from 10^7^ to 1×10^1^ nominal copy equivalent/reaction. Copy number of test samples was determined by interpolation of the experimentally determined C_T_ value for the test sample onto the control standard regression curve. Calculated copy equivalent per reaction values was then normalized and expressed as copy equivalents per milliliter of starting plasma. Assay was accepted for r^2^ value of the standard curve being >0.98.

### Computational analysis of GP sequences

Multiple alignment of Ebola glycoprotein (GP) sequences (Zaire 1976, GenBank Accession No. NC_002549; Bundibugyo, Accession No. FJ217161; Sudan 2000, Accession No. NC_006432) was performed with the program ClustalW2 available at the EBI server (http://www.ebi.ac.uk/Tools/clustalw2/).

The article "Demonstration of Cross-Protective Vaccine Immunity against an Emerging Pathogenic Ebolavirus Species" was published in 2010. Journal: PLoS Pathog.

To model the molecular relationship between the glycoprotein of the vaccine strain (Zaire Mayinga 1976) and of the virus infecting strain (Bundibugyo 2007), an alignment was generated by using the program MAFFT [31] and improved manually. The GP amino acid sequences included in this alignment were Ebola Zaire Mayinga 1976 (Accession No. Q05320), Zaire Ekron 1976 (Accession No. P87671), Sudan Boniface 1976 (Accession No. Q66814), Sudan Maleo 1979 (Accession No. Q66798), Gabon 1994/1997 (Accession No. AAC57989 and O11457), Sudan Gulu (Accession No. Q7T9D9), Zaire Kikwit 1995 (Accession No. P87666), Reston (Accession No. Q66799), Cote d'Ivoire (Accession No. Q66810), and Bundibugyo 2007 (Accession No. ACI28624). A distance-based phylogenetic analysis was performed using the programs in the PHYLIP 3.68 package [32]. The distance matrix was calculated using the Jones-Taylor-Thornton (JTT) substitution model [33]. These distances were clustered with the neighbor-joining (NJ) algorithm [34]. Five hundred nonparameteric bootstrap replicates were performed to assess support for individual clades by the data. In the figure the numbers at the nodes of the tree are the bootstrap percentages, where any value greater than 0.70 indicates strong support for that grouping in the data. Branch lengths are measured in substitutions per site. The multiple sequence alignment was also analyzed using parsimony with the program PAUP. Five heuristic searches, each with an independent random starting tree, were performed and a consensus of the most parsimonious tree or trees from these searches was calculated. Five hundred nonparametric bootstrap replicates were performed to assess the support of the trees by the data. Bootstrap percentages are indicated at the nodes of the tree and are interpreted as for the distance analysis.

### Statistics

Differences in survival outcome were compared by log rank test using GraphPad Prism 5.0 software. Averaged data values are presented as mean ± SEM. Comparison of anti-Ebola GP antibody titers (EC90) and intracellular cytokine production by T cell memory subsets were done using one-tailed T-test in GraphPad software.

### Ethics statement

The authors have declared that no competing interests exist. All animal experiments were conducted under protocols approved by NIH and USAMRIID Animal Care and Use committees. All animal experiments were conducted under protocols approved by NIH and USAMRIID Animal Care and Use committees. All experiments involving the use of BEBOV in animals were performed in USAMRIID's BSL-4 laboratory. Research was conducted in compliance with the Animal Welfare Act and other federal statutes and regulations relating to animals and experiments involving animals and adheres to principles stated in the Guide for the Care and Use of Laboratory Animals, National Research Council, 1996. The facility where this research was conducted is fully accredited by the Association for Assessment and Accreditation of Laboratory Animal Care International. Animals were housed individually, and given enrichment regularly as recommended by the Guide for the Care and Use of Laboratory Animals (DHEW number NIH 86-23).
